# The Efficacy and Safety of Acupuncture in the Treatment of Neurodermatitis: A Systematic Review and Meta-Analysis

**DOI:** 10.1155/2022/8182958

**Published:** 2022-09-01

**Authors:** Lin Yang, Xinyun Li, Wei Huang, Jialiang Li, Xiangshu Rao, Yu Lai

**Affiliations:** ^1^School of Basic Medicine, Chengdu University of Traditional Chinese Medicine, Chengdu 611137, China; ^2^School of Traditional Chinese Medicine, Sichuan College of Traditional Chinese Medicine, Mianyang, China

## Abstract

**Background:**

Neurodermatitis is a common chronic inflammatory skin disease associated with neurological dysfunction. This study aimed to explore the efficacy and safety of acupuncture and moxibustion in the treatment of neurodermatitis through meta-analysis.

**Methods:**

We comprehensively searched 9 databases, including PubMed, Cochrane Library, EMBASE, Web of Science, Scopus, China National Knowledge Infrastructure (CNKI), Wanfang Database, China Science and Technology Journal Database (VIP), and China Biomedicine (CBM), from their inception to November 15, 2021, for published neurological and clinical randomized controlled trials (RCTs) using acupuncture to treat dermatitis. We also searched gray literature in four databases: Chinese Clinical Trials Registry, Chinese Cochrane Center, Open Grey, and GreyNet International. Two authors independently screened the data, extracted the literature, and evaluated the quality of the literature using Cochrane 5.3.3 and Review Manager 5.4.1 software.

**Results:**

The meta-analysis included 8 studies with a total of 728 participants, including 369 patients in the treatment group and 359 patients in the control group. Compared with conventional treatment, acupuncture significantly increased the effective rate (OR: 2.90, 95% CI: 1.78∼4.75; *p* < 0.001) and decreased the recurrence rate after treatment (OR: 0.26, 95% CI: 0.12∼0.59; *p*=0.001). Meanwhile, analysis of disease symptom scores showed that acupuncture group had a greater impact (OR: 3.51, 95% CI: 2.12∼4.91; *p* < 0.00001). Furthermore, no significant difference in the adverse reaction rate was observed.

**Conclusion:**

Acupuncture is safe and effective in treating neurodermatitis. However, the current level of research evidence is limited, and therefore, larger sample and high-quality RCTs are needed to confirm its safety and effectiveness. Protocol registration number is INPLASY2021110041.

## 1. Introduction

Neurodermatitis is a common chronic inflammatory skin disease associated with neurological dysfunction, paroxysmal itching, and lichen-like skin changes. Scratching and friction are important factors leading to lichenoid changes in this disease [1]. The incidence of the disease is approximately 12%, and women are more likely to develop this disease than men [2, 3]. This disease causes psychosocial burdens on patients and sleep disorders and affects the quality of work and quality of life of patients [4]. The cause of this disease is currently unclear, although it is generally believed that the disease may be caused by cerebral cortex or excitatory dysfunction [5]. Moreover, several internal and external factors, such as mental stress, anxiety, depression, local irritation, and endocrine disorders, may also affect neurodermatitis [6–9]. Clinical treatments usually include glucocorticoids, antihistamines, antidepressants, local immunomodulators, and other drugs [10, 11]. However, the curative effects are unsatisfactory, and the condition readily recurs after cessation of drug treatment. In addition, long-term use of hormone drugs is associated with a series of complications, such as telangiectasia, osteoporosis, local skin atrophy, and other adverse reactions [12, 13]. Therefore, other treatments that can reduce itching and lichen-like changes in the skin of patients with neurodermatitis have attracted increasing attention.

Acupuncture is a component of traditional Chinese medicine that has long existed in our history and has gradually gained widespread and global recognition due to its safety, effectiveness, and reliability [14, 15]. Dozens of studies have suggested that acupuncture could be used to treat many skin diseases [16–18]. Several studies have suggested that acupuncture can reduce the release of itch mediators such as histamine and 5-hydroxytryptamine (5-HT), thereby reducing the intensity of itch-related diseases [3, 19–21]. Moreover, acupuncture can also improve the lichen-like symptoms of neurodermatitis [3]. However, the available body of research lacks uniform efficacy standards and high-quality randomized controlled trials (RCTs); thus, it has been impossible to comprehensively and objectively evaluate the efficacy of acupuncture in treating neurodermatitis.

In the present study, we conducted a systematic review and meta-analysis to evaluate the effectiveness and safety of acupuncture in the treatment of neurodermatitis. Our study involved different forms of acupuncture, such as needle, skin needle (inserting short needles into the superficial part of the body), electroacupuncture (a small amount of pulse current is passed through the needle), fire needle (a method of rapidly piercing acupoints with a red-hot needle to treat diseases), warm needle (a kind of therapy that uses acupuncture while adding warm stimulation), and moxibustion (a method of stimulating human acupoints with heat produced by moxa strips or columns made of moxa leaves). Our purpose was to select RCTs with similar characteristics evaluating acupuncture and moxibustion in the treatment of neurodermatitis through uniform inclusion criteria to clarify the effectiveness and safety of acupuncture and moxibustion in the treatment of neurodermatitis. All these efforts could provide a valuable evidence-based foundation to guide clinical and medical practice.

## 2. Methods

### 2.1. Study Registration

The meta-analysis was based on the Cochrane Handbook for Systematic Reviews of Interventions (5.3.3) and the Preferred Reporting Items guidelines for System reviews and Meta-Analysis using Review Manager. This protocol was registered in the International Platform of Registered Systematic Review and Meta-analysis Protocols. The register name is “Effectiveness of Acupuncture in the Treatment of Neurodermatitis: A Systematic Review and Meta-Analysis.” The registration number was INPLASY2021110041.

### 2.2. Ethics

Since the systematic review was based on published research, it did not require the approval of an ethics committee.

### 2.3. Search Strategy

We searched the following 9 electronic databases (5 English databases and 4 Chinese databases): PubMed, Cochrane Library, EMBASE, Web of Science, Scopus, China National Knowledge Infrastructure (CNKI), Wanfang Database, China Science and Technology Journal Database (VIP), and China Biomedicine (CBM) from their inception to 15 November 2021. In addition, gray literature from the China Clinical Trials Registry, Chinese Cochrane Center, Open Grey, and GreyNet International from their inception to November 15, 2021, was also searched [22]. This study considered RCTs of acupuncture treatment of neurodermatitis, and there were no language restrictions implemented in the search. The search strategy used a combination of subject terms and free words. Based on the characteristics of each database, the search strategy was as follows: (“acupuncture” [MeSH] OR “electro acupuncture” [Title/Abstract] OR “fire needle” [Title/Abstract] OR “moxibustion” [Title/Abstract] OR “cutaneous acupuncture” [Title/Abstract] OR “warm needle acupuncture” [Title/Abstract] OR “needle” [Title/Abstract]) AND (“Neurodermatitis” [MeSH] OR “Neurodermatitides” [Title/Abstract] OR “Lichen Simplex Chronicus” [Title/Abstract] OR “Neurodermatitis, Localized” [Title/Abstract] OR “Localized Neurodermatitides” [Title/Abstract] OR “Localized Neurodermatitis” [Title/Abstract] OR “Neurodermatitides, Localized” [Title/Abstract] OR “Neurodermatitis, Circumscribed” [Title/Abstract] OR “Circumscribed Neurodermatitides” [Title/Abstract] OR “Circumscribed Neurodermatitis” [Title/Abstract] OR “Neurodermatitides, Circumscribed” [Title/Abstract]).  Table 1 shows the PubMed search strategy as an example.

### 2.4. Eligibility Criteria

#### 2.4.1. Inclusion Criteria

(1) Participants. Subjects were clinically diagnosed with neurodermatitis. There were no restrictions on the patients' age, sex, country, or ethnicity. (2) Study types: only RCTs written in Chinese or English were included. (3) The following intervention types were considered: needle, fire needle, electric acupuncture, skin needle, and other types of acupuncture, regardless of the choice of acupoints and Chinese medicine treatment. The control group was treated with conventional drugs or for symptoms. (4) Main outcomes: the effective rate, recurrence rate, disease change score, and adverse reaction rate were assessed.

#### 2.4.2. Exclusion Criteria

(1) Duplicate publications and studies with incomplete data were excluded. (2) Reviews, theoretical discussions, animal experiments, meeting minutes, and nonrandomized controlled experiments were excluded. (3) Studies including pregnant and lactating women were excluded. (4) Treatment groups using traditional Chinese medicine or acupuncture and other drugs in combination were excluded; control groups were treated with acupuncture and moxibustion-related treatments.

### 2.5. Outcome Measurements

The outcome measurements included the effective rate, recurrence rate, changes in disease symptom score, and adverse reaction rate.

### 2.6. Study Selection

All studies were entered in Endnote and independently screened by two authors (Lin Yang and Xinyun Li). The two authors manually deleted studies with duplicate titles and abstracts. After excluding duplicate studies, preliminary screening was conducted by reading the titles and abstracts to exclude nonconforming studies based on research type, participants, and interventions. Then, after reviewing the full text, studies that met the inclusion criteria were included. In the process of study selection, any disagreements were resolved through consultation with the third author (Jialiang Li).

### 2.7. Data Extraction

The data were independently extracted by two authors (Lin Yang and Xinyun Li). The extracted data were cross-checked for a final determination of data integrity and authenticity. The extracted content included author, publication year, sample size, male-to-female ratio, age of research subjects, research method, intervention measures used in each group, treatment time, and outcome indicators. If the results were inconsistent, any differences were resolved through consultation with the third author (Jialiang Li).

### 2.8. Bias Risk Assessment

Two authors (Lin Yang and Xinyun Li) independently assessed the quality of each study. The Cochrane Handbook for Systematic Reviews of Interventions and RevMan 5.4 software were used to evaluate the quality of the included studies. The quality evaluation of 7 areas for each study included the following: random sequence generation, allocation concealment, blinding of participants and personnel, blinding of outcome assessment, incomplete outcome data, selective reporting, and other bias. The risk of bias was classified as “low risk,” “unclear risk,” or “high risk.” If the results were inconsistent, any differences were resolved through consultation with the third author (Xiangshu Rao).

### 2.9. Data Analysis

RevMan 5.4 software downloaded from the Cochrane website was used to analyze the data included in the literature. Stata software version 16.0 was used to perform funnel chart analyses and sensitivity analyses. The odds ratios (ORs) and the 95% credible intervals (CIs) were selected as the statistics with binary data. Continuous variables are represented by mean differences (MDs) and 95% confidence intervals. The Cochrane chi-square test and *I*^2^ were used to test heterogeneity between studies. When *I*^2^ > 50% and *I*^2^ < 50%, we used a random effects model and fixed effects model, respectively, to summarize the data. Funnel charts were used to assess whether there was potential publication bias, and *p* < 0.05 was considered to be significantly different. Sensitivity analyses were used to evaluate the robustness and reliability of the research.

## 3. Results

### 3.1. Study Selection

Based on the search strategy, a total of 1301 articles were retrieved from the establishment of the database to November 15, 2021. In the process of searching for gray literature, no suitable or valuable literature was obtained [22]. Then, we manually deleted 597 duplicate articles. There were 696 remaining articles that were excluded because they did not meet our inclusion criteria. For example, the article was a review or a theoretical discussion, there was no full text, or the use of acupuncture was combined with drug treatment. Two authors independently screened the articles based on the inclusion and exclusion criteria. In summary, 8 articles were included in this meta-analysis [1, 23–29] (Figure 1). A total of 728 patients were randomly assigned to the treatment group (*n* = 369) and control group (*n* = 359).

### 3.2. Basic Characteristics of the Included Studies

A total of 728 patients were studied in these 8 studies, including 369 patients in the treatment group and 359 patients in the control group. All 8 RCTs were conducted in China. The studies reported general information such as age and length of intervention. The sample size of each group was between 26 and 94 participants. The treatment cycle for the treatment group and the control group was between 2 weeks and 1 month. 3 studies in the treatment group used fire needle treatment [1, 25, 29], and 5 studies used skin acupuncture plus moxibustion treatment [23, 24, 26–28]. The control group used conventional drug intervention. Eight studies reported on the effectiveness. 5 studies reported the recurrence rate after treatment [24–27, 29]. 2 studies showed changes in the disease symptom score [24, 26]. 2 studies reported adverse reactions [25, 26]. The characteristics of the study are shown in Tables 2 and 3.

### 3.3. Bias Risk Assessment

8 studies included in this meta-analysis were RCTs. 1 study [29] used a high-risk random method. The bias risk of 2 studies [26, 27] was not clear because they did not mention the specific method of random sequence generation. 2 studies [23, 24] using statistical software for random allocation and three studies [1, 25, 28] using random number tables were all low risk. Only one study [23] mentioned the application of allocation concealment-related information, and the other studies did not describe allocation concealment. Regarding performance bias, one study [26] mentioned nonblinding.

Only one study [26] mentioned blinding of outcome assessment, and the other studies did not clearly describe whether blinding was used for result measurement. The bias risk of all trials was rated low risk regarding outcome completeness. The bias risk of all trials was rated low risk regarding selective reporting. Due to insufficient information, other biases were classified as unclear risk. The specific risk deviation assessment is shown in Figures 2 and 3.

### 3.4. Results of the Meta-Analysis

#### 3.4.1. Effective Rate

Effectiveness is the main result of this research. The effectiveness of the 8 studies was evaluated after treatment. A total of 728 patients were studied. Among them, the treatment group included 369 patients, and 359 patients were studied in the control group. The statistics showed that the *I*^2^ heterogeneity was 8%, and the *p* value of the *χ*^2^ test was 0.37 (*p* > 0.1). There was no obvious heterogeneity among these studies; thus, the fixed effects model was used. The results showed that the effective rate in the acupuncture group was significantly higher than that in the control group (OR: 2.90, 95% CI: 1.78∼4.75; *p* < 0.001). The combined statistical test (*Z* = 4.25 and *p* < 0.0001) was statistically significant (Figure 4). There was no significant heterogeneity among these studies, and therefore, no subgroup analysis was performed.

#### 3.4.2. Recurrence Rate

5 studies [24–27, 29] reported the recurrence rate of patients in the treatment group and the control group. Statistical analysis showed that there was no obvious heterogeneity between the treatment group and the control group (*I*^2^ = 0% and *p*=0.98). Therefore, the fixed-effects model was applied to analyze the effect of acupuncture on the treatment of neurodermatitis (Figure 5). The results showed that there was a significant difference in the recurrence rate between the acupuncture group and the control group. The recurrence rate in the acupuncture group was lower than that in the control group (OR: 0.26, 95% CI: 0.12∼0.59; *p*=0.001).

#### 3.4.3. Changes in Disease Symptom Scores

2 studies [24, 26] compared changes in disease symptom scores before and after treatment. A total of 178 patients in 2 studies included 92 patients in the treatment group and 86 patients in the control group. *I*^2^ = 0% and *p*=0.95 indicated that there was no obvious heterogeneity between these studies; thus, the fixed effects model was used for further analysis. The difference between the treatment group and the control group was statistically significant (OR: 3.51, 95% CI: 2.12∼4.91; *p* < 0.00001). The results showed that the acupuncture group had significantly lower disease symptom scores (Figure 6).

#### 3.4.4. Safety Analysis

2 studies [25, 26], which included 85 patients in the treatment group and 83 patients in the control group, reported the adverse effects of acupuncture in the treatment of neurodermatitis. The fixed effect model was used for analysis due to no obvious heterogeneity between the studies (*I*^2^ = 0% and *p*=0.33) (Figure 7). The data showed that, in terms of adverse reactions, there was no significant difference between the acupuncture group and the control group (OR: 0.32, 95% CI: 0.05∼2.05; *p*=0.23).

### 3.5. Publication Bias

We conducted funnel plot analyses with the effective rate of the eight RCTs to analyze publication bias. According to the funnel plot, the effective rate was asymmetrically distributed (Figure 8(a)). In Begg's test, the *p* value of the effective rate was 0.108 (*p* > 0.05). Meanwhile, the recurrence rate distribution was symmetrical (Figure 8(b)). In Begg's test, the *p* value of the effective rate was 0.806 (*p* > 0.05). Since the number of included studies for other outcomes was too small (*n* < 5), funnel plots were not constructed.

### 3.6. Sensitivity Analysis

Through the sensitivity analysis of the effective rate and recurrence rate of the study, after converting the effect model or excluding the results of the included studies one by one, the effect size of the outcome indicators did not significantly change, and the results were the same as the original conclusion. Efficient sensitivity analysis showed that the lowest and highest values of the confidence interval were 1.51 and 6.18, respectively. The meta-analysis effect size of the efficient sensitivity analysis showed that the upper and lower limits of the confidence interval were 1.78 and 4.75, respectively. Sensitivity analysis of the recurrence rate showed that the lowest and highest values of the confidence interval were 0.13 and 0.75, respectively. Meanwhile, the meta-analysis effect size results of the sensitivity analysis showed that the upper and lower limits of the confidence intervals were 0.17 and 0.61, respectively. Sensitivity analysis proved that this study has good stability.

### 3.7. Trial Sequential Analysis

We implemented trial sequential analysis (TSA) (version 0.9.5.10 Beta) software to perform the trial sequential analysis. Our study set a 5% risk of type I error and a relative risk reduction of 20% (power of 80%) to evaluate the required information size (RIS) and the trial sequential monitoring boundary (TSMB). If the cumulative *Z*-value crosses the TSMB and RIS threshold, the sample size is sufficient. The results on the effective rate and recurrence rate were considered reliable and stable because the *Z*-value crossed the trial sequential monitoring boundary and required information size. The results showed that the acupuncture group was more effective in treating neurodermatitis than the control group, while the recurrence rate of the acupuncture group was lower than that of the control group (Figures 9(a) and 9(b)).

## 4. Discussion

Neurodermatitis is a clinically common chronic inflammatory skin disease involving nerve dysfunction; however, conventional drug treatment of this disease is not ideal. Therefore, other effective treatment methods are very important. In this systematic review and meta-analysis, a total of 8 studies and 728 patients were included (369 patients in the treatment group and 359 patients in the control group). Our research showed that acupuncture was better than conventional drugs in the treatment of neurodermatitis. The results showed that acupuncture significantly improved the effective rate and reduced the recurrence rate. Research data have found that the acupuncture group had a greater impact on changes in disease symptom scores from before to after treatment. However, in terms of safety, there was no significant difference between the acupuncture group and the control group.

Through the collected data, we found that acupuncture can effectively treat neurodermatitis, although the level of evidence is not high. Itching is the most important clinical manifestation of neurodermatitis. Itching can affect people's work, life, and rest, and the itching-scratching cycle can not only aggravate itching but also lead to lichen-like changes in the skin. Itching stems from the activation of peripheral nerve endings after injury or exposure to inflammatory mediators [30]. In the skin, itch is mainly transmitted by C-fibers and thinly myelinated type A*δ* nerve fibers [31]. Acupuncture stimulates C-fibers to induce the expansion of peripheral blood vessels and quickly consume neurotransmitters, thereby achieving antipruritic effects [32]. Carlsson et al. reported that acupuncture can interfere with the transmission of central and peripheral itching, which may help reduce itching [32]. In addition, skin lichenification is another important manifestation of neurodermatitis. Dozens of studies have found that acupuncture can improve local microcirculation, speed up metabolism, strengthen fiber cell regeneration, reduce local inflammation, and promote the repair of damaged tissues [3, 33, 34]. Neuroimaging data have shown that acupuncture can regulate a wide range of brain regions, such as limbic, prefrontal, and brainstem regions, which is a possible mechanism for acupuncture to treat skin itching [35]. Thus, acupuncture stimulates the body's benign self-adjustment, regulates the body's functions, improves the body's internal environment, improves mental states, and relieves symptoms such as anxiety, thereby achieving the effect of curing neurodermatitis [36, 37].

Our meta-analysis also showed that acupuncture can effectively reduce the recurrence rate of neurodermatitis. Neurodermatitis is a common recurring skin disease [12]. The recurrence rate of the disease can increase in the case of mental stress, anxiety, work stress, endocrine disorders, and so on. In this study, acupuncture treatment was better than control treatment in reducing the recurrence rate. This may be because acupuncture can stimulate the body's self-adjustment and relieve anxiety. Therefore, compared with other treatments, acupuncture can reduce the recurrence rate of neurodermatitis. This can not only reduce a patient's physical and mental pain and economic burden but also reduce the social burden and save medical resources.

The analysis of disease symptom scores suggested that the acupuncture group scores were greater than the control group scores. However, in this meta-analysis, only 2 studies reported disease symptom scores before and after treatment. Therefore, reporting bias cannot be ruled out. In clinical practice, stronger evidence is needed to prove this hypothesis.

In terms of the safety of acupuncture, there was no significant difference between the acupuncture group and the control group. It was found that needle fainting occurred in the acupuncture group, which subsided after rest [26]. In the control group, mild gastrointestinal discomfort and aggravation of symptoms occurred after treatment [25, 26]. In particular, there were no serious adverse events in the acupuncture group or the control group. In short, this study shows to a certain extent that acupuncture is a safe and effective treatment for neurodermatitis. In terms of the safety analysis, there was no significant difference between the two experimental groups, suggesting that more research is needed to explore the safety of acupuncture in the future.

This study has some strengths. This meta-analysis suggests that acupuncture can be used as a beneficial auxiliary treatment method, which can reduce the use of hormonal drugs, thereby reducing the recurrence rate and adverse reactions. No systematic reviews of acupuncture for neurodermatitis have been published in the past decade. Previous systematic reviews have mainly focused on a single type of intervention or acupuncture combined with other drugs or treatments to treat neurodermatitis [38, 39]. Our main focus was on the effects of common forms of acupuncture, which reduced the introduction of possible variability due to including other forms of acupuncture. This approach can more accurately evaluate the role of acupuncture in the treatment of neurodermatitis.

Future research needs to establish more rigorous experimental designs to improve the quality of the experimental research; for example, allocation concealment and blinding can be implemented. All the studies in this meta-analysis were conducted in China, and participants can be recruited from other countries for RCTs of acupuncture and moxibustion in the treatment of neurodermatitis.

Notably, this study has several limitations. First, the number and sample size of the included studies were relatively small. There is a lack of high-quality, large-sample clinical RCTs, resulting in the poor research level of this meta-analysis. Second, the included studies were all from China, which may have increased the heterogeneity among the included studies and may have limited the generalizability to patients in other countries and regions. Third, due to the particularities of acupuncture, there are certain difficulties regarding allocation concealment and blinding methods in the experimental design, so the included studies may have been biased. In addition, only 2 studies reported adverse reactions to acupuncture in the treatment of neurodermatitis, so the analysis of safety results may have been limited. Finally, the selection of acupuncture points and acupuncture stimulation used across the studies included in this analysis may have been different, which is not conducive to a unified analysis.

In conclusion, acupuncture can be used as an important supplementary and alternative treatment method for treating neurodermatitis because it can effectively improve clinical symptoms and reduce recurrence. In the future, high-quality RCTs with large-sample sizes are needed to confirm the results discussed in this systematic review.

## 5. Conclusions

This systematic review and meta-analysis found that acupuncture can effectively and safely treat neurodermatitis by significantly improving the effective rate, reducing the recurrence rate, and changing the disease symptom scores. However, due to the current low-level quality of the evidence, future high-quality, large-sample size randomized controlled experiments are needed to further confirm this conclusion.

## Figures and Tables

**Figure 1:** A flowchart showing the selection process.

**Figure 2:** Diagram of the bias risk.

**Figure 3:** Summarized risk of bias.

**Figure 4:** Forest plot for effective rate between the experimental and control groups.

**Figure 5:** Outcomes of the meta-analysis for the influence of acupuncture on recurrence rate.

**Figure 6:** Forest graph of the changes in disease symptom score.

**Figure 7:** Forest plot shows the safety comparison between the acupuncture group and the control group.

**Figure 8:** Publication bias.

**Figure 9:** Results of required information size (RIS) with acupuncture treatment variant: (a) effective rate for experiment vs. control;(b) recurrence rate for experiment vs. control. The required information size was calculated based on a two-sided *α* = 5%, *β* = 15% (power 80%), and a relative risk reduction of 20%.

**Table 1:** PubMed search strategy.

Number	Search terms
^#^21	^#^8 AND ^#^20
^#^20	^#^9 OR ^#^10 OR ^#^11 OR ^#^12 OR ^#^13 OR ^#^14 OR ^#^15 OR ^#^16 OR ^#^17 OR ^#^18 OR ^#^19
^#^19	“Neurodermatitides, circumscribed” [title/abstract]
^#^18	“Circumscribed neurodermatitides” [title/abstract]
^#^17	“Neurodermatitides, localized” [title/abstract]
^#^16	“Localized neurodermatitides” [title/abstract]
^#^15	“Neurodermatitis, localized” [title/abstract]
^#^14	“Neurodermatitides” [title/abstract]
^#^13	“Circumscribed neurodermatitis” [title/abstract]
^#^12	“Neurodermatitis, circumscribed” [title/abstract]
^#^11	“Localized neurodermatitis” [title/abstract]
^#^10	“Lichen simplex chronicus” [title/abstract]
^#^9	“Neurodermatitis” [mesh]
^#^8	^#^1 OR ^#^2 OR ^#^3 OR ^#^4 OR ^#^5 OR ^#^6 OR ^#^7
^#^7	“Cutaneous acupuncture” [title/abstract]
^#^6	“Needle” [title/abstract]
^#^5	“Warm needle acupuncture” [title/abstract]
^#^4	“Moxibustion” [title/abstract]
^#^3	“Fire needle” [title/abstract]
^#^2	“Electro acupuncture” [title/abstract]
^#^1	“Acupuncture” [mesh]

**Table 2:** Characteristics information of the included studies.

Author	Country	Year	Sample size	I	C	I	C
				Sex (M/F)	Sex (M/F)	Age (year)	Age (year)
Yunkuan Yang	China	2006	54	9/19	11/15	38.86 ± 14.46	40.38 ± 15.61
Jishu Li	China	2007	80	—	—	38.24 ± 13.67	36.00 ± 13.91
Zhen Tian	China	2015	70	—	—	25–50	25–50
Yan Li	China	2016	60	17/13	10/20	36.98 ± 9.04	34.12 ± 10.34
Zhan Wang	China	2008	98	23/27	25/23	37.26 ± 11.84	38.48 ± 10.54
Canyang Diao (1)	China	2007	120	29/31	34/26	18–65	19–63
Canyang Diao (2)	China	2007	60	17/13	16/14	18–65	19–63
Hongfei Ci	China	2015	186	38/56	41/51	48.3 ± 10.6	46.4 ± 12.7

I = intervention; C = control; M = male; F = female; A = acupuncture; M = medicine.

**Table 3:** Characteristics information of the included studies.

Author	Year	I	C	Treatment cycle	I	C
					Treatment frequency	Treatment frequency
Yunkuan Yang	2006	A	M	1 month	Once every 2 days	3 times a day
Jishu Li	2007	A	M	1 month	Once every 2 days	3 times a day
Zhen Tian	2015	A	M	1 month	Once every 7 days	2 times a day
Yan Li	2016	A	M	1 month	Once every 2-3 days	2 times a day
Zhan Wang	2008	A	M	1 month	Once every 2 days	3 times a day
Canyang Diao (1)	2007	A	M	1 month	Once every 2 days	3 times a day
Canyang Diao (2)	2007	A	M	1 month	Once every 2 days	3 times a day
Hongfei Ci	2015	A	M	2 weeks-1 month	2 times a week	1-2 times a day

I = intervention; C = control; M = male; F = female; A = acupuncture; M = medicine.

## Data Availability

The table data used to support the findings of this study are included within the article. The figure data used to support the findings of this study are included within the figure files.
